# Intelligent Optimization Algorithm-Based Path Planning for a Mobile Robot

**DOI:** 10.1155/2021/8025730

**Published:** 2021-09-29

**Authors:** Qisong Song, Shaobo Li, Jing Yang, Qiang Bai, Jianjun Hu, Xingxing Zhang, Ansi Zhang

**Affiliations:** ^1^School of Mechanical Engineering, Guizhou University, Guiyang 550025, Guizhou, China; ^2^State Key Laboratory of Public Big Data, Guizhou University, Guiyang 550025, Guizhou, China; ^3^School of University South Carolina, Department of Computer Science and Engineering, Columbia, SC 29201, USA

## Abstract

The purpose of mobile robot path planning is to produce the optimal safe path. However, mobile robots have poor real-time obstacle avoidance in local path planning and longer paths in global path planning. In order to improve the accuracy of real-time obstacle avoidance prediction of local path planning, shorten the path length of global path planning, reduce the path planning time, and then obtain a better safe path, we propose a real-time obstacle avoidance decision model based on machine learning (ML) algorithms, an improved smooth rapidly exploring random tree (S-RRT) algorithm, and an improved hybrid genetic algorithm-ant colony optimization (HGA-ACO). Firstly, in local path planning, the machine learning algorithms are used to train the datasets, the real-time obstacle avoidance decision model is established, and cross validation is performed. Secondly, in global path planning, the greedy algorithm idea and B-spline curve are introduced into the RRT algorithm, redundant nodes are removed, and the reverse iteration is performed to generate a smooth path. Then, in path planning, the fitness function and genetic operation method of genetic algorithm are optimized, the pheromone update strategy and deadlock elimination strategy of ant colony algorithm are optimized, and the genetic-ant colony fusion strategy is used to fuse the two algorithms. Finally, the optimized path planning algorithm is used for simulation experiment. Comparative simulation experiments show that the random forest has the highest real-time obstacle avoidance prediction accuracy in local path planning, and the S-RRT algorithm can effectively shorten the total path length generated by the RRT algorithm in global path planning. The HGA-ACO algorithm can reduce the iteration number reasonably, reduce the search time effectively, and obtain the optimal solution in path planning.

## 1. Introduction

Path planning is an important research direction in the field of mobile robots, which has become a powerful promoter in the era of digital economy. Path planning is the most important research field of mobile robots [1]. The definition of path planning is to find a collision-free path from the starting point to the target point according to some related performance indicators (such as time, distance, energy consumption, and real-time performance) in a multiobstacle environment. Its goal is to find an optimal path with the least time, the shortest path, the least energy consumption, and the strongest real-time performance.

Path planning is mainly divided into local path planning [2] and global path planning [3] according to the degree of environmental cognition. Path planning algorithms are mainly divided into classical intelligent optimization algorithm [4] and heuristic intelligent optimization algorithm [5] according to the era of algorithm research.

The following problems need to be resolved in the path planning at the current stage. The mobile robot has poor real-time obstacle avoidance performance in local path planning, the accuracy of real-time obstacle avoidance needs to be improved, it is easy to fall into the local optimum, and the overall path planning efficiency is not high. Meanwhile, the mobile robot has poor search efficiency in global path planning, time-consuming is longer, prone to collision, and the path cannot reach optimum. In addition, path planning algorithms have poor versatility, local path planning algorithms have poor performance in global path planning, and global path planning algorithms have poor performance in local path planning.

In order to improve the accuracy of real-time obstacle avoidance of mobile robots in local path planning and obtain a collision-free safe path, improve the path optimization performance of mobile robot in global path planning and effectively shorten the path length, enhance the versatility of the path planning algorithm, and make the mobile robot obtain an optimal path with shorter time-consuming and more accurate obstacle avoidance in local and global path planning, therefore, this paper performs corresponding optimization research on path planning algorithms.

The main contributions of this paper are described as follows:

1. A real-time obstacle avoidance decision model based on machine learning algorithms is designed to improve the accuracy and speed of real-time obstacle avoidance prediction for mobile robots in local path planning.
2. A new improved S-RRT algorithm is proposed to smooth the global path and shorten the total length of the path, which introduces the greedy algorithm idea and B-spline curve into the RRT algorithm and can remove the redundant nodes of path.
3. A new HGA-ACO algorithm is proposed to shorten the path length and time and generate a more stable collision-free optimization path. It is based on the idea of hybrid algorithm, combines the advantages of genetic algorithm and ant colony optimization, and can generate better paths in global path planning and local path planning.

The main organizational structure of this paper is as follows: Section 2 mainly describes the related work of intelligent optimization algorithm for path planning.  Section 3 mainly introduces local path planning based on machine learning algorithms and establishes a real-time obstacle avoidance decision model.  Section 4 describes the global path planning based on the S-RRT algorithm and introduces the overall optimization process of the S-RRT algorithm.  Section 5 describes the path planning based on HGA-ACO and introduces the optimization process and fusion strategy of genetic algorithm and ant colony optimization.  Section 6 summarizes our contributions and draws some future research lines.

## 2. Related Work

The classical intelligent optimization algorithm includes RRT, artificial potential field (APF), dynamic window approach (DWA), and differential evolution (DE) [6]. The heuristic intelligent optimization algorithm includes genetic algorithm (GA), Ant colony optimization (ACO), and particle swarm optimization (PSO) [7].

For classical intelligent optimization algorithms, Fan et al. [8] proposed the improved APF applied for autonomous underwater vehicle, which solved the problem of path target unreachable. Chang et al. [9] proposed an improved DWA, which improved the success rate of paths in unknown environment by optimizing and adding evaluation functions. Hu et al. [10] proposed an efficient RRT-based framework to generate shorter and smoother paths with less computation. Qi et al. [11] proposed a MOD-RRT*∗*, which is composed of path generation and path planning, and it is suitable for robot navigation in unknown dynamic environment. In addition, researchers have also performed more optimization studies on the RRT algorithm, such as DT-RRT [12], Bidirectional RRT*∗* [13], and PQ-RRT*∗* [14].

For heuristic intelligent optimization algorithms, Nazarahari et al. [15] applied an enhanced GA to multiobjective multirobot path planning in continuous environment. Hao et al. [16] proposed an adaptive genetic algorithm based on collision detection, which solves the problem of low quality of genetic algorithm paths and low convergence iterations by optimizing genetic operators and adding collision detection methods. Ma et al. [17] proposed a genetic algorithm based on Bezier curves, which can effectively generate shorter and smoother paths. Li et al. [18] proposed an improved ACO, which improved the convergence speed by adaptively changing the wave coefficient and updating the state transition rules. Miao et al. [19] proposed an improved adaptive ant colony algorithm, which balances the convergence problem through adaptive adjustment factors to obtain a more stable path. Xie et al. [20] proposed a mixed cognition PSO, which calculated fitness through minimum-maximum normalization and transformed the multiobjective path optimization problem into a single-objective path optimization problem. Xiong et al. [21] applied the improved A ^*∗*^ algorithm to intelligent vehicle trajectory planning, which improved the accuracy of path tracking. The improved fuzzy logic algorithm is applied to vehicle and UAV path planning, which improves the stability and real-time performance of the path [22].

Now, researchers have proposed many hybrid algorithms based on the coevolution strategy [23], such as hybrid genetic artificial neural network algorithm [24] and hybrid Genetic and Fuzzy logic algorithms [25]. Ravankar et al. [26] proposed a hybrid potential based probabilistic roadmap algorithm, which improved the efficiency of the algorithm and can generate paths in narrow channels. Wang et al. [27] proposed a hybrid genetic tabu search algorithm for two-stage path planning and real-time path trajectory control of mobile robot in automatic storage retrieval system. Chen et al. [28] proposed a bidirectional A*∗* algorithm based on ant colony algorithm, which effectively shortened the path search time and enhanced the dynamic search ability. Peng et al. [29] proposed the chaos-based PSO-ACO, which has a rapid path search speed and can be applied for harsh environments such as deep sea or coal mine.

It can be seen from the above research that other methods of path planning at this stage are to optimize the single type of local or global paths. The method proposed in this paper fully considers the local and global paths and carries out the corresponding optimization research on these two types of common algorithms, and the overall research on path planning is more comprehensive.

RRT algorithm is a classical algorithm of global path planning algorithm, which can be applied to any type of mobile robot. It has a fast path optimization speed and has a great research prospect in global path planning. HGA-ACO algorithm is a hybrid optimization algorithm of GA and ACO. It makes full use of the global search performance of GA and the strong robustness of ACO, which can speed up the convergence speed and generate a smoother and more stable optimal path.

In addition, different path planning algorithms have their own limitations, a single type of path planning algorithm cannot obtain an ideal path in complex environments, and multiple path planning algorithms can obtain ideal paths in complex environments and promote the development of path planning research. Therefore, this paper focuses on S-RRT algorithm and HGA-ACO algorithm.

## 3. Machine Learning Algorithm

### 3.1. Machine Learning Introduction

Local path planning is a kind of online path planning applied in unknown and complex environment, which needs to continuously collect surrounding environment information and provide timely feedback. Therefore, good real-time obstacle avoidance performance is the research focus of local path planning, and the use of machine learning algorithms [30] can improve the real-time obstacle avoidance ability of mobile robots in complex unknown environments and can accurately determine the moving direction. Machine learning algorithms mainly include Multinomial Naive Bayesian (MNB), Gaussian Naive Bayesian (GNB), Support Vector Machines (SVM), K-Nearest Neighbor (KNN), and Random Forests (RF).

The NB classification model can be expressed by the following equation:

(1) $$\begin{array}{c} P\left(c|x\right)=\frac{P\left(c\right)*P\left(x|c\right)}{P\left(x\right)}=\frac{P\left(x,c\right)}{P\left(x\right)}, \end{array}$$

where *P*(*c|x*) is posteriori probability, *P*(*x*, *c*) is conditional probability, and *P*(*x*) and *P*(*c*) are priori probabilities.

The SVM classification model can be expressed by equation (2) or equation (3) according to whether the training set is linearly separable.

(2) $$\begin{array}{c} \left\{\begin{array}{c} X_{i}+b\geq 1,\;\forall X_{i}\in P,\\ W^{t}X_{i}+b\geq -1,\;\forall X_{i}\in N,\\ f_{w,b}\left(X\right)=\mathrm{sgn}\left(W^{t}X_{i}+b\right), \end{array}\right. \end{array}$$

(3) $$\begin{array}{c} L\left(w\right)=\frac{\left\|\overset{⟶}{w}\right\|}{2}+C\left(\sum_{i=1}^{N}\xi_{i}^{k}\right), \end{array}$$

where *W*^*t*^ is the weight parameter, *b* is the bias parameter, and *L*(*w*) is the Lagrange function.

The Euclidean Distance formula used in the KNN classification model can be expressed by equations (4) and (5):

(4) $$\begin{array}{c} d\left(p,q\right)=\sqrt{\sum_{i=1}^{n}{\left(p_{i}-q_{i}\right)}^{2}}, \end{array}$$

(5) $$\begin{array}{c} W=\frac{1}{d{\left(p,q\right)}^{2}}, \end{array}$$

where *p*_*i*_ and *q*_*i*_ are two eigenvalues, *n* is the characteristic dimension, and *W* is the weight factor.

The RF classification model can be expressed by the following equation:

(6) $$\begin{array}{c} f\left(x\right)=\mathrm{mod}e\left(T_{1}\left(x\right),\ldots ,T_{n}\left(x\right)\right), \end{array}$$

where *T* is the decision tree and *n* is the number of decision trees.

### 3.2. Obstacle Avoidance Dataset

The obstacle avoidance data comes from the open dataset of University of California Irvine at https://archive.ics.uci.edu/ml/datasets/Wall-Following+Robot+Navigation+Data. The data were collected as the SCITOS G5 robot navigates through the room following the wall in a clockwise direction, for 4 rounds. The “simplified distance” is composed of the minimum readings of the distance to the obstacle detected by the ultrasonic sensor within its 60° arc.

Taking “simplified distance” as the characteristic value and the robot moving direction as the label value, the characteristic values mainly include front, left, right, and behind distance. The label values mainly include Move-Forward, Slight-Right Turn, Sharp-Right Turn, and Slight-Left Turn. Preprocess the obstacle avoidance dataset, and then describe it in the form of characteristic values and label values, as shown in Figure 1.

It can be seen from Figure 1 that when the front distance is large, the direction of obstacle avoidance movement of the robot is Move-Forward; when the right distance is large, the direction of obstacle avoidance movement of the robot is Sharp-Right Turn; when the front distance and the right distance are large, the direction of obstacle avoidance movement of the robot is Slight-Right Turn; when the front distance and the left distance are large, the direction of obstacle avoidance movement of the robot is Slight-Left Turn.

### 3.3. Real-Time Obstacle Avoidance Decision Model

For the robot obstacle avoidance dataset, different ML algorithms are used to train the sample data, generate a real-time obstacle avoidance decision model, and make predictions on the sample data. The dataset has a total of 5456 data, where 1636 are training samples, and 3820 are test samples. By comparing the prediction results with the actual sample data, the prediction performance of various ML algorithms can be judged. The evaluation standard for the performance of ML algorithms is comprehensive evaluation index, which includes accuracy, precision, recall, F1-Measure, and Mcc. Confusion matrix is a visualization tool for comprehensive evaluation index, as shown in Table 1.

From Table 1, we can see what is the relationship between actual and forecast, and then, we can get formulas for comprehensive evaluation index. Accuracy, precision, recall, F1-Measure, and Mcc can be expressed by equations (7)–(11), respectively:

(7) $$\begin{array}{c} \text{Accuracy}=\frac{\text{TP}+\text{TN}}{\text{TP}+\text{TN}+\text{FP}+\text{FN}}, \end{array}$$

(8) $$\begin{array}{c} \text{Precision}=\frac{\text{TP}}{\text{TP}+\text{FP}}, \end{array}$$

(9) $$\begin{array}{c} \text{Recall}=\frac{\text{TP}}{\text{TP}+\text{FN}}, \end{array}$$

(10) $$\begin{array}{c} F1=\frac{2*\text{Precision}*\text{Recall}}{\text{Precision}+\text{Recall}}, \end{array}$$

(11) $$\begin{array}{c} \text{Mcc}=\frac{\text{TP}*\text{TN}-\text{FP}*\text{FN}}{\sqrt{\left(\text{TP}+\text{FP}\right)*\left(\text{TP}+\text{FN}\right)*\left(\text{TN}+\text{FP}\right)*\left(\text{TN}+\text{FN}\right)}}, \end{array}$$

where TP is True Positive, FN is False Negative, FP is False Positive, TN is True Negative, Accuracy is the proportion of samples that are correctly classified, Precision is the proportion of true positive samples in the recognized positive samples, Recall is the proportion of samples recognized as positive in the total positive samples, F1 is the harmonic average of precision and recall, and Mcc is the correlation coefficient between the predicted result and the actual result.

The aim of this work is to propose a real-time obstacle avoidance decision model through machine learning algorithms to improve the real-time obstacle avoidance prediction performance of mobile robots in local path planning. The steps involved are as follows:

1. Collecting and preprocessing obstacle avoidance dataset
2. Dividing the dataset into training sample dataset and test sample dataset
3. Training process: training sample dataset through the ML algorithm classifier to establish a real-time obstacle avoidance decision model
4. Testing process: the real-time obstacle avoidance decision model is used to predict the test sample dataset and analyze the predictive performance
5. Tenfold cross-validation is used to improve the accuracy and obtain a more stable and reliable model

### 3.4. Simulation Experiments

The trained real-time obstacle avoidance decision model is used to predict the sample data, and then the prediction results are obtained. The fitting curve between the actual data and the prediction results is shown in Figure 2.

After the dataset is preprocessed, the label values are converted; that is, Move-Forward, Slight-Right Turn, Sharp-Right Turn, and Slight-Left Turn are converted to 0, 1, 2, and 3, respectively. The *x*-axis and *y*-axis in Figure 2 represent the number and the label value of test dataset, respectively. The blue curve represents the actual result, and the pink curve in 2(a), the yellow curve in 2(b), and the red curve in 2(c) represent the prediction results of NB, SVM, and RF, respectively. It can be seen from Figure 2 that the predicted result of RF is almost completely fitted with the actual result, while the fitting effect of other machine learning algorithms is poor. It indicates that RF has the best predictive effect compared with other machine learning algorithms.

In order to analyze the prediction performance of the real-time obstacle avoidance decision model established by the machine learning algorithm, the comprehensive evaluation index is used to show the model effect. The experimental results of the comprehensive evaluation index are shown in Figure 3.

It can be seen from Figure 3 that the comprehensive evaluation index of the RF has reached 99.9%, while the comprehensive evaluation indexes of KNN, SVM, GNB, and MNB are about 95.5%, 93.7%, 89.7%, and 58.7%, respectively. Therefore, the RF has the highest overall performance, followed by KNN, SVM, and GNB, and MNB is the lowest.

In order to prevent overfitting caused by the complexity of real-time obstacle avoidance decision model, the tenfold cross-validation is introduced to test the accuracy of the algorithm. The experimental results of the tenfold cross-validation comprehensive evaluation index are shown in Figure 4.

It can be seen from Figure 4 that the comprehensive evaluation index of the RF has reached 99.8%, while the comprehensive evaluation indexes of KNN, SVM, GNB, and MNB are about 93.2%, 91.5%, 88.4%, and 58.3%, respectively. Although the comprehensive evaluation index of the machine learning algorithm after tenfold cross-validation is slightly lower than before, a more reliable and stable model can be obtained.

## 4. S-RRT Algorithm

### 4.1. S-RRT Introduction

The traditional RRT algorithm is a sampling-based global path planning algorithm that takes the starting point as the algorithm root node and continuously expands new leaf nodes until the end point is found. It will randomly generate many scattered nodes, and the path is not smooth enough. In view of the problem of unsmooth global path, the improved S-RRT algorithm is proposed to smooth the global path, so as to obtain a shorter and smoother path. The principle of the improved S-RRT algorithm is to introduce the idea of greedy algorithm on the basis of the RRT algorithm, divide the growing tree in the state space into several subgrowing trees, first find out the local optimal solution of each subgrowing tree, and then synthesize the multiple local optimal solution into the global optimal solution.

The improved S-RRT algorithm mainly consists of two parts: the first part is the improved RRT algorithm, and the second part is the smooth RRT algorithm. *T*, *p*, *q*, *X*_init_, *X*_near_, *X*_rand_, *X*_target_, *X*_goal_, and *X*_parent_ represent the random tree, the probability threshold, the random probability value, the initial state point, the nearest state point, the random state point, the target state point, the goal state point, and the parent state point in the configuration space, respectively.

### 4.2. S-RRT Process

Generally speaking, the improved RRT algorithm can be summarized in Algorithm 1. In Algorithm 1, the path target state point is determined by setting the probability threshold and comparing the probability threshold with the random probability value. If *q* > *p*, it means that the exploring random tree will regard *X*_goal_ as *X*_target_, else *q* < *p*, the exploring random tree will regard *X*_rand_ as *X*_target_. Introducing the idea of variable probability target bias can reduce the expansion of random nodes and speed up the expansion of nodes to goal.

The proposed smooth RRT algorithm can be illustrated in Algorithm 2. In Algorithm 2, in order to solve the problem of redundant nodes in the RRT algorithm, the denoising operation based on the principle of internode connectivity is adopted to delete all redundant nodes not on the RRT path. Then, use the idea of greedy algorithm [31] to divide the exploring random tree into subexploring random trees, regard the initial state point as the starting point of the subexploring random tree, and use the reverse retrospective mechanism to update the parent state point until the collision-free parent state point connected to the initial state point is found, and it is used as the goal point of the subexploring random tree. As for the smoothness of the path, the B-spline curve is used to smooth the path nodes to ensure the continuity of the path curvature.

The B-spline curve has the advantages of continuity and local adjustability [32]. Therefore, the S-RRT algorithm makes full use of the advantages of the B-spline curve to fit the global path generated by the RRT algorithm to generate a smooth path with continuous curvature, which can ensure the continuity and smoothness of the mobile robot motion.

The expression of k-order B-spline curve can be written as the following equation:

(12) $$\begin{array}{c} P\left(u\right)=\sum_{i=0}^{n}P_{i}*N_{i,K}\left(u\right), \end{array}$$

where *P*_*i*_ is the control point, *n* is the number of control points, and *N*_*i*,*K*_(*u*) is the basis function of the K-order B-spline curve.

The B-spline curve basis function is a k-order piecewise polynomial determined by a sequence of nondecreasing parameters of a node vector, that is, a k-order polynomial spline. It can be obtained by Cox-de Boor recurrence relation and can be written as equations (13) and (14):

(13) $$\begin{array}{c} N_{i,0}\left(u\right)=\left\{\begin{array}{cc} 1, & u_{i}\leq u\leq u_{i+1},\\ 0, & \text{otherwise,} \end{array}\right. \end{array}$$

(14) $$\begin{array}{c} N_{i,k}\left(u\right)=\frac{u-u_{i}}{u_{i+k}-u_{i}}N_{i,k-1}\left(u\right)+\frac{u_{i+k+1}-u}{u_{i+k+1}-u_{i+1}}N_{i+1,k-1}\left(u\right), \end{array}$$

where *N*_*i*,0_(*u*) is the basis function of the 0-order B-spline curve and *N*_*i*,*k*−1_(*u*) is the basis function of the *k* − 1-order B-spline curve.

In order to obtain *N*_*i*,*K*_(*u*), a total of *k* + 1 parameter nodes are required such as *u*_*i*_, *u*_*i*+1_,…, *u*_*i*+*k*_; therefore, [*u*_*i*_, *u*_*i*+*k*_] is called the support interval of *N*_*i*,*K*_(*u*). For a K-order B-spline curve and *n* + 1 control points, the union of support intervals defines a set of B-spline basis node vector *T* =[*u*_0_, *u*_1_,…, *u*_*n*_,…, *u*_*n*+*k*_]. In order to meet the constraints of the starting and the target state, the curve must go through the starting and the target point. The nodes at both ends of the sample have the degree of repetition *k*, which means that the node vector must satisfy the following equation:

(15) $$\begin{array}{c} \left\{\begin{array}{c} u_{0}=u_{1}=\cdots =u_{k},\\ u_{n}=u_{n+1}=\cdots =u_{n+k}, \end{array}\right. \end{array}$$

where *u* is node vector and *u*_*k*_ is the *k*th node vector.

### 4.3. Simulation Experiments

In order to prove the superiority of the improved S-RRT algorithm, the simulation for the global path planning of mobile robots is carried out to compare the improved S-RRT algorithm with the RRT algorithm. The size of the whole state space is 20 cm × 20 cm, the black rectangular frames are obstacle regions, the fixed step *δ* is 1.7 cm, and the probability threshold *p* is 0.6. One experimental path for RRT in three experimental scenarios is shown in the green lines of Figures 5(a), 5(c), and 5(e), respectively. Figures 5(b), 5(d), and 5(f) give the final generated smooth path (shown in the red line) for the improved S-RRT algorithm. It can be seen from Figure 5 that the smooth path generated by the S-RRT algorithm is shorter than RRT algorithm.

Taking into account the randomness of the RRT algorithm and the objective evaluation of its performance, 20 path planning experiments are carried out with two algorithms in three experimental scenarios, respectively. The comparison of the pathing length from the two algorithms in three scenarios is shown in Figure 6(a) and marked by a different color and line style. Additionally, Figures 6(b) and 6(c) also give the comparison of the pathing nodes and running time from the two algorithms in three scenarios. Then, the average pathing length and pathing nodes as well as the running time are recorded, respectively, and are shown in Table 2.

From the related data in Figure 6 and Table 2 of the simulation experiment, the conclusion can be drawn that the pathing length and pathing nodes with S-RRT are improved better than RRT. Furthermore, the paths are smoother and can avoid the obstacle completely, which meet the requirement of smooth motion for the mobile robot in the process of obstacle avoidance.

## 5. HGA-ACO

### 5.1. Problem Definition

Path planning is a multiobjective optimization problem [33], which needs to consider the safety, smoothness, and total length of the path. Its mathematical model is as follows, where formula (16) represents the safety of the minimized path, formula (17) represents the smoothness of the minimized path, and formula (19) represents the length of the minimized path:

(16) $$\begin{array}{c} \min f_{1}\left(P\right)=-\underset{0\leq i\leq n}{\min}\underset{1\leq j\leq m}{\min}\left\{D_{\min}\left(\bar{p_{i}p_{i+1}},O_{j}\right)\right\}, \end{array}$$

(17) $$\begin{array}{c} \min f_{2}\left(P\right)=\frac{1}{n}\sum_{i=0}^{n-1}\left(\pi -\;\cos^{-1}\left(\delta \right)\right), \end{array}$$

(18) $$\begin{array}{c} \delta =\frac{\left(x_{i+1}-x_{i}\right)\left(x_{i+2}-x_{i+1}\right)+\left(y_{i+1}-y_{i}\right)\left(y_{i+2}-y_{i+1}\right)}{d\left(p_{i},p_{i+1}\right)d\left(p_{i+1},p_{i+2}\right)}, \end{array}$$

(19) $$\begin{array}{c} \min f_{3}\left(P\right)=\sum_{i=0}^{n-1}\sqrt{{\left(x_{i+1}-x_{i}\right)}^{2}+{\left(x_{i+2}-x_{i}\right)}^{2}}, \end{array}$$

where *P* is the path, *p*_*i*_ is the *i*th node of the path, its coordinates are (*x*_*i*_, *y*_*i*_), *O*_*j*_ is the *j*th obstacle, $\bar{p_{i}p_{i+1}}$ is the road segment between the node *i* and node *i* + 1, *δ* is the cosine value of the corners of two adjacent road segments, and *d*(*p*_*i*_, *p*_*i*+1_) is the distance between two adjacent path nodes.

The mathematical model simplifies the complex path planning problem into a mathematical problem, which makes the problem description more scientific, logical, and objective, and then facilitates the quantitative analysis of the path planning problem.

### 5.2. HGA-ACO Process

The proposed HGA-ACO combines the advantages of GA and ACO and can be applied to both local path planning and global path planning. It not only optimizes the path but also eliminates algorithmic barriers, providing a reference for the integration of multiple algorithms. The construction of the HGA-ACO in path planning is shown in Figure 7.

### 5.3. Optimizing GA

#### 5.3.1. Optimizing Fitness Function of GA

The fitness function is the decisive factor in the genetic algorithm to determine whether to reach the optimal path. Therefore, improving the traditional fitness function is the most important task of path optimization. The optimized fitness function we proposed is based on the fitness function of genetic algorithm and introduces the fitness function of path smoothness, which can make the path generated by the robot smoother.

Fitness function of genetic algorithm: the reciprocal of the total length from the start point to the end point of the path. Fitness function can be written as the following equation:

(20) $$\begin{array}{c} f_{1}=\frac{1}{\sum_{i=1}^{n-1}\sqrt{{\left(x_{i+1}-x_{i}\right)}^{2}+{\left(y_{i+1}-y_{i}\right)}^{2}}}, \end{array}$$

where *f*_1_ is the fitness function of genetic algorithm and *x*_*i*_ and *y*_*i*_ are the values of the *X* coordinate axis and *Y* coordinate axis of the nodes *i*, respectively.

Fitness function of path smoothness: the reciprocal of the sum of path penalty coefficients.

First, calculate the distance between two adjacent nodes and three adjacent nodes. These distances can be written as equations (21) and (22):

(21) $$\begin{array}{c} d_{1i}=\sqrt{{\left(x_{i+1}-x_{i}\right)}^{2}-{\left(y_{i+1}-y_{i}\right)}^{2}},\;i\in \left(1,n-1\right), \end{array}$$

(22) $$\begin{array}{c} d_{2i}=\sqrt{{\left(x_{i+2}-x_{i}\right)}^{2}-{\left(y_{i+2}-y_{i}\right)}^{2}},\;i\in \left(1,n-2\right), \end{array}$$

where *n* is the total number of nodes in the path and *d*_1*i*_ and *d*_2*i*_ are the distances between any two and three adjacent nodes in the path, respectively.

Then, judge the included angle between three adjacent nodes according to the node distance. The included angle can be written as the following equation:

(23) $$\begin{array}{c} \theta =\left\{\begin{array}{cc} 45^{{}^{\circ}}, & d_{1i}=1,\;d_{2i}=1\cap d_{1i}=\sqrt{2},\;d_{2i}=1,\\ 90^{{}^{\circ}}, & d_{1i}=1,\;d_{2i}=\sqrt{2}\cap d_{1i}=\sqrt{2},\;d_{2i}=2,\\ 135^{{}^{\circ}}, & d_{1i}=1,\;d_{2i}=2\cap d_{1i}=\sqrt{2},\;d_{2i}=\sqrt{5},\\ 180^{{}^{\circ}}, & d_{1i}=1,\;d_{2i}=\sqrt{5}\cap d_{1i}=\sqrt{2},\;d_{2i}=2\sqrt{2}, \end{array}\right. \end{array}$$

where *θ* is the included angle between three adjacent nodes in the path, which are determined by the value of *d*_1*i*_ and *d*_2*i*_.

In addition, the corresponding penalty coefficients are introduced to the included angles according to the robot kinematics and dynamics constraints. The penalty coefficients can be written as the following equation:

(24) $$\begin{array}{c} w_{k}=\left\{\begin{array}{cc} 0, & \theta =45^{{}^{\circ}},\\ 10. & \theta =90^{{}^{\circ}},\\ 100, & \theta =135^{{}^{\circ}},\\ 10000, & \theta =180^{{}^{\circ}}, \end{array}\right. \end{array}$$

where *w*_*k*_ is the penalty coefficients, which is judged by the value of *θ*.

Finally, the sum of the penalty coefficients corresponding to the angles of all nodes of the overall path is calculated. The fitness function of path smoothness can be written as the following equation:

(25) $$\begin{array}{c} f_{2}=\frac{1}{\sum_{k=1}^{n-2}w_{k}}, \end{array}$$

where *f*_2_ is the fitness function of path smoothness.

Optimize fitness function: under the corresponding weight coefficients, the sum of the fitness function of genetic algorithm and the fitness function of path smoothness. First, introduce the corresponding weight coefficient to the fitness function of the genetic algorithm and fitness function of the path smoothness, respectively. Then, the fitness functions under the weight coefficients are added. The larger the weight coefficient corresponding to the fitness function of path length and path smoothness, the greater the influence on the optimize fitness function. The optimize fitness function can be written as the following equation:

(26) $$\begin{array}{c} f=a*f_{1}+b*f_{2}, \end{array}$$

where *f* is the optimize fitness function and *a* and *b* are the weight coefficients corresponding to the fitness function of genetic algorithm and the fitness function of path smoothness, respectively.

#### 5.3.2. Optimizing Genetic Operation Method of GA

After optimizing the fitness function, there are many excellent individuals in the next generation, and complex elite retention mechanism is not needed. The selection method we adopt is probability-based roulette, which guarantees that some of the best individuals of the offspring are retained, maintains the diversity of the population, and avoids falling into the local optimum. The probability of individual fitness function can be written as the following equation:

(27) $$\begin{array}{c} P_{i}=\frac{f_{i}}{\sum_{i=1}^{n}f_{i}}, \end{array}$$

where *f*_*i*_ is the optimal fitness function of individuals in the population and *P*_*i*_ is the probability of individual optimized fitness function in the population.

The crossover method we adopt is a single-point crossover optimization method, which is divided into two categories according to whether the crossover genes are the same. The first type is the single-point crossover method without the same gene number (seen in Figure 8(a)), it randomly selects a different gene as a crossover point, and they exchange genes after that point with each other. The second type is the single-point crossover method with the same gene number (seen in Figure 8(b)), and it randomly selects the same gene as a crossover point, and they exchange genes after that point with each other.

The single-point crossover optimization method selects the best individuals from the parent and offspring to enter the next generation, avoiding population degradation caused by the traditional single-point crossover.

The mutation method we adopt is a multidirectional mutation method, which is divided into two categories according to the direction of mutation (see in Figure 9). The mutation individual is selected according to the mutation probability, and then the mutation points are randomly selected from them.

The first type takes the mutation point as the starting point and the *S* point as the end point to perform reverse search to obtain the mutated individuals, and the second type takes *G* point as the starting point and the mutation point as the end point to perform reverse search to obtain the mutated individuals. By comparing the fitness of the two mutated individuals, the individual with higher fitness was selected. It means that the robot generates more optimal paths in path planning and prevents the path from developing in a worse direction.

### 5.4. Genetic-Ant Colony Fusion Strategy

The pheromone accumulation optimization strategy we adopted is to import the optimized path of the genetic optimization algorithm into the ant colony algorithm; it is a key step in the fusion of genetic optimization algorithm and ant colony optimization algorithm. By making full use of the strong global search ability of genetic algorithm, the multiple optimization paths generated by genetic algorithm are introduced into ant colony algorithm to become its initial pheromone. In this way, HGA-ACO can skip the initial pheromone accumulation stage of the ant colony algorithm, so as to solve the problem of the lack of pheromone in the initial stage of the ant colony algorithm and shorten the pheromone accumulation time. Among them, the multiple optimization paths generated by the genetic optimization algorithm are selected according to the fitness value of the last generation individual, and the part of individuals with a larger fitness value is continuously selected as the initial pheromone of the ant colony algorithm. The specific conversion steps are as follows:

1. Select some individuals with larger fitness values in the last generation generated in the genetic optimization algorithm
2. The acquired individuals form a matrix *T*
3. Traverse each row of the matrix *T* and convert it into a pheromone value according to the conversion formula
4. Initialize the converted pheromone value

The conversion formula can be written as the following equation:

(28) $$\begin{array}{c} \tau_{ij}=\tau_{ij}^{g}=\tau_{ji}^{g}=\frac{\varphi }{D_{T_{n}}*l_{ij}}, \end{array}$$

where *τ*_*ij*_ is the initial pheromone value from node *i* to node *j* in the grid map; *τ*_*ij*_^*g*^ and *τ*_*ji*_^*g*^ are the initial pheromone values of ant colony algorithm, which is converted from the partial optimal path between node *i* and node *j* generated by genetic optimization algorithm; *T*_*n*_ is a matrix *T* composed of partially optimized paths; *D*_*T*_*n*__ is the path length corresponding to the part of the individual converted into the initial pheromone in the genetic optimization algorithm, that is, the length of the partial optimal path; *l*_*ij*_ is the straight line distance between node *i* and node *j*; *φ* is a constant.

### 5.5. Optimizing ACO

#### 5.5.1. Optimizing Pheromone Update Strategy of ACO

The basic principle of pheromone update [34] in ant colony algorithm is to use different state transition probabilities to determine the choice of the next node according to the different pheromone concentrations in the surrounding feasible regions, which leads to continuous changes in the pheromone concentration. The original state transition probability can be written as equations (29) and (30):

(29) $$\begin{array}{c} P_{ij}^{k}\left(t\right)=\left\{\begin{array}{cc} \frac{\tau_{ij}^{\alpha }\left(t\right)*\eta_{ij}^{\beta }\left(t\right)}{\sum_{k\in N_{k}}\tau_{ik}^{\alpha }\left(t\right)*\eta_{ik}^{\beta }\left(t\right)}, & k\in N_{k},\\ 0, & k\notin N_{k}, \end{array}\right. \end{array}$$

(30) $$\begin{array}{c} \eta_{ij}=\frac{Q}{d_{ij}}, \end{array}$$

where *P*_*ij*_^*k*^(*t*) is the selection probability of ants moving from node *i* to node *j* at time *t*; *τ*_*ij*_^*α*^(*t*) is the pheromone concentration between node *i* and node *j* at time *t*; *η*_*ij*_^*β*^(*t*) is the heuristic information between node *i* and node *j* on the feasible path at time *t*, that is, the degree of expectation; *α* is pheromone heuristic factor; *β* is the expectation heuristic factor; *N*_*k*_ is the set of next feasible nodes that individual *k* can choose at node *i*.

By optimizing the pheromone update method of the MAX-MIN Ant System, it not only retains the advantages of its global optimal path update, but also introduces the update of the current iterative optimal path, which realizes the update of the current and global optimal paths and avoids the loss of the remaining optimal paths in the iteration.

In the optimization of the pheromone update strategy, corresponding weights are set for the current iterative optimal path and the global optimal path respectively, and the sum of the two weights is the maximum number of iterations. The weight of the current iterative optimal path is set to the maximum number of iterations during the initialization of the algorithm. As the HGA-ACO continues to iteratively optimize, the weight of the current iterative optimal path continues to decrease, while the weight of the global optimal path continues to increase. It means that the pheromone concentration of the global optimal path is enhanced in the iterative update, and the optimized pheromone update strategy can more accurately find the optimal path. The optimized pheromone update rules can be written as equations (31)–(33):

(31) $$\begin{array}{c} \tau_{ij}\left(t+1\right)=\left(1-\rho \right)*\tau_{ij}\left(t\right)+\Delta \tau_{ij}\left(t\right), \end{array}$$

(32) $$\begin{array}{c} \Delta \tau_{ij}\left(t\right)=\left(\frac{A}{D_{g}}+\frac{B}{D_{n}}\right)*\frac{1}{N_{c}}, \end{array}$$

(33) $$\begin{array}{c} A+B=N_{c}, \end{array}$$

where *ρ* is the pheromone evaporation rate, Δ*τ*_*ij*_(*t*) is the increment of pheromone at time *t*, *τ*_*ij*_(*t*) is the pheromone value at time *t*, *τ*_*ij*_(*t*+1) is the pheromone value at time *t* + 1, *A* is the weight of the global optimal path, *B* is the weight of the current iterative optimal path, *D*_*g*_ is the total length of the global optimal path, *D*_*n*_ is the total length of the current iterative optimal path, and *N*_*c*_ is the maximum number of iterations.

The above is HGA-ACO's pheromone update optimization method for the better path. Of course, for the poor path generated in the algorithm, the optimized pheromone update method is also adopted, and its goal is to make the poor path pheromone dissipate continuously with iterative updates. The optimized pheromone update rules for poor paths can be written as the following equation:

(34) $$\begin{array}{c} \tau_{ij}\left(t+1\right)=\left(1-\rho \right)*\tau_{ij}\left(t\right), \end{array}$$

where *τ*_*ij*_(*t*) is the pheromone value at time *t* and *τ*_*ij*_(*t*+1) is the pheromone value at time *t* + 1.

Compared with the better path, its optimization strategy lacks the pheromone increment, which means that the pheromone has been evaporating instead of accumulating. Therefore, HGA-ACO will not choose these poor paths when planning the path, so as to realize the continuous optimization of the path and avoid the generation of poor paths.

#### 5.5.2. Deadlock Elimination Strategy

The deadlock problem is that the ant colony algorithm encounters concave obstacles in the path planning, which makes it unable to plan the next node. Its appearance has caused great troubles to the path planning for ant colony algorithm, reducing the speed of convergence and wasting running time. In response to the deadlock problem, HGA-ACO develops a deadlock elimination strategy; that is, a penalty function is introduced to establish a dead-angle table. The dead-angle table is composed of the deadlock points in the environment map, the deadlock points are the position points when entering the deadlock state, and the path planning for HGA-ACO will not go to any deadlock points in the dead-angle table. The introduction of the penalty function can reduce the pheromone concentration at the edge of the dead-angle in the environmental map, instruct HGA-ACO to avoid the edge of the dead-angle as much as possible during the next iteration, speed up the path optimization process, reduce the number of iterations, and eliminate deadlock problems. The penalty function can be written as the following equation:

(35) $$\begin{array}{c} \tau \left(i,j\right)=\lambda *\tau \left(i,j\right),\;0<\lambda <1, \end{array}$$

where *λ* is the penalty coefficient, and the value range is 0 to 1, and *τ*(*i*, *j*) is the pheromone concentration at the edge of the dead-angle.

### 5.6. Simulation Experiments

In order to prove the advantage and validity of the HGA-ACO algorithm, the simulation for the global path planning of mobile robots is carried out to compare it with ACO and GA. The size of the grid map is 20 cm × 20 cm, the black rectangular frames are obstacle regions, and the parameter settings in the HGA-ACO are as follows: *P*_c_=0.8, *P*_m_=0.2, *a*=1, *b*=7, *N*_*c*_=100, *M*=50, *ρ*=0.3, *Q*=1, *α*=1, *β*=7, *N*_max_=100, *A*=0, and *B*=100.

The simulation experiments are carried out with three algorithms in three experimental scenarios, respectively.  Figure 10 gives the robot path trajectory for HGA-ACO (shown in the red line), the robot path trajectory for ACO (shown in the blue line), and the robot path trajectory for GA (shown in the green line). The simulation results for HGA-ACO, ACO, and GA in scenario 1, scenario 2, and scenario 3 are shown in Figures 10(a)–10(c), Figures 10(d)–10(f), and Figures 10(g)–10(i), respectively. It can be seen from Figure 10 that the robot path trajectory generated by HGA-ACO is the shortest and the smoothest.

The comparison of the iteration curve from the three algorithms in three scenarios is shown in Figure 11(a)-c and marked by a different color and line style. Additionally, the path length and running time as well as the optimal iteration are recorded, respectively, and are shown in Table 3.

From the related data in Figure 11 and Table 3 of the simulation experiment, the conclusion can be drawn that the HGA-ACO has the shortest path length, the shortest running time, the minimum iteration numbers, and the fastest convergence. The proposed HGA-ACO is superior to GA and ACO in terms of search speed, optimization efficiency, and accuracy, which is proved to be a successful algorithm.

## 6. Conclusions

In the local path planning, we have proposed a real-time obstacle avoidance decision model established by machine learning algorithm, which can improve the accuracy of the path real-time obstacle avoidance prediction. Among the machine learning algorithms, RF has the best prediction performance, and the prediction accuracy is almost 99.9%.

In the global path planning, we have proposed an improved S-RRT algorithm based on the idea of greedy algorithm and the B-spline curve. Compared with the RRT algorithm, the improved S-RRT algorithm can shorten the path length, improve the search efficiency, and reduce the path redundant points effectively, and the generated paths are much smoother.

In the path planning, we have proposed a HGA-ACO algorithm combined with the improved GA and the improved ACO, which makes full use of the global optimization ability of genetic algorithm and the robustness of ant colony algorithm. It can optimize the local path in real time on the basis of generating the global optimization path and then obtain the global optimal path. Compared with GA and ACO, it has a shorter path length, less running time, and fewer optimal iterations. Most importantly, the proposed HGA-ACO can be applied to local and global path planning, and its path planning performance exceeds other related path planning algorithms mentioned in this paper.

In this paper, we have proposed powerful methods for robot path planning, which achieved good results in simulation and improved the overall performance of path planning. In the future, we will verify our proposed method in actual working conditions and study new intelligent optimization algorithms.

## Figures and Tables

**Figure 1:** The robot obstacle avoidance dataset.

**Figure 2:** Fitting curve of machine learning.

**Figure 3:** Comprehensive evaluation index.

**Figure 4:** Tenfold cross validation.

**Figure 5:** Robot path trajectory for RRT/S-RRT. (a) Initial path generated by the RRT in scenario 1; (b) smooth path generated by the S-RRT in scenario 1; (c) initial path generated by the RRT in scenario 2; (d) smooth path generated by the S-RRT in scenario 2; (e) initial path generated by the RRT in scenario 3; (f) smooth path generated by the S-RRT in scenario 3.

**Figure 6:** Comparison of the two algorithms in three scenarios. (a) Comparison of the pathing length; (b) comparison of the pathing nodes; (c) comparison of the running time.

**Figure 7:** Flowchart of HGA-ACO in path planning.

**Figure 8:** Single-point crossover optimization method.

**Figure 9:** Multidirectional mutation method.

**Figure 10:** Robot path trajectory for HGA-ACO/ACO/GA. (a) Robot path trajectory for HGA-ACO in scenario 1; (b) robot path for ACO in scenario 1; (c) robot path for GA in scenario 1; (d) robot path for HGA-ACO in scenario 2; (e) robot path for ACO in scenario 2; (f) robot path for GA in scenario 2; (g) robot path for HGA-ACO in scenario 3; (h) robot path for ACO in scenario 3; (i) robot path for GA in scenario 3.

**Figure 11:** Iteration curve from the three algorithms in three scenarios. (a) Iteration curve from the three algorithms in scenario 1; (b) iteration curve from the three algorithms in scenario 2; (c) iteration curve from the three algorithms in scenario 3.

**Algorithm 1:** Algorithm 1 Improved RRT.

**Algorithm 2:** Algorithm 2 Smooth RRT.

**Table 1:** Confusion matrix.

Prediction		
Real	Positive	Negative
Positive	TP	FP
Negative	FN	TN

**Table 2:** Simulation comparison result of different algorithms.

	Scenario 1			Scenario 2			Scenario 3		
Algorithm	Average pathing length (cm)	Average pathing nodes	Average running time (s)	Average pathing length (cm)	Average pathing nodes	Average running time (s)	Average pathing length (cm)	Average pathing nodes	Average running time (s)
S-RRT	30.27	4.25	1.7816	30.47	3.35	2.1130	30.90	4.35	2.2260
RRT	36.50	20.5	1.4617	35.33	20.05	1.7116	36.64	20.70	1.8562

**Table 3:** Simulation comparison result of different algorithms.

	Scenario 1			Scenario 2			Scenario 3		
Algorithm	Path length (cm)	Running time (s)	Optimal iteration	Path length (cm)	Running time (s)	Optimal iteration	Path length (cm)	Running time (s)	Optimal iteration
HGA-ACO	28.6274	1.36	10	29.7990	1.49	2	29.2132	1.42	20
ACO	29.4558	14.76	65	31.4558	15.27	68	29.2132	14.33	50
GA	30.6274	2.83	36	30.2132	2.51	33	30.3848	2.57	28

## Data Availability

The data used to support the findings of this study are included within the paper. All required models and parameters are listed in the paper.
